# The ING4 Binding with p53 and Induced p53 Acetylation were Attenuated by Human Papillomavirus 16 E6

This article has been retracted.

**DOI:** 10.1371/journal.pone.0071453

**Published:** 2013-08-13

**Authors:** Yi Guo, Xiangkai Meng, Qian Wang, Yanan Wang, Hong Shang

**Affiliations:** 1 Department of Gynecology, First Affiliated Hospital of China Medical University, Shenyang, China; 2 Key Laboratory of AIDS Immunology of Ministry of Health, Department of Laboratory Medicine, First Affiliated Hospital of China Medical University, Shenyang, China; Vanderbilt University Medical Center, United States of America

## Abstract

High risk subtype HPV16 early oncoprotein E6 contributes host cell immortalization and transformation through interacting with a number of cellular factors. ING4 is one member of the inhibitor of growth (ING) family of type II tumor suppressors and it has been shown to be involved in regulating p53 function. However, the effect and mechanism of HPV16 E6 on ING4 function remain elusive. In this study, we report HPV16 E6 combines with ING4 in vivo and in vitro. The ING4 induced p53 acetylation and its combining with p53 were attenuated by HPV16 E6 independent of p53 degradation. The enhancing function of ING4 on p53 mediated apoptosis was diminished when HPV16 E6 existed. These findings reveal that ING4 may be a common target of oncogenic viruses for driving host cell carcinogenesis.

## Introduction

It is well known that the high risk type of human papillomaviruses (HPVs) are etiological agents in cervical carcinogenesis [1], [2]. HPV16 early proteins E6 and E7 are the major oncoproteins which are crucial for host cell immortalization and transformation by inactivating the tumor suppressors, p53 and pRB, respectively [3]. Furthermore, inhibition of E6/E7 expression impedes the growth of HPV positive cancer cells [4]. Particularly, E6 recruits a ubiquitin protein ligase E6AP, and the resulted complex targets the p53 tumor suppressor protein for proteasome mediated degradation [5], [6]. E6AP is also important for E6 mediated degradation of other cellular partners such as hScribble, a PDZ domain partner [7], hMCM7 [8], E6TP1 [9], and Myc [10] which is involved in activation of TERT [11]. However, E6 also can inactivate p53 independently of E6AP [12], [13]. Besides E6AP, HPV16 E6 interacts with several other cellular proteins, including ATF3 [14], E6BP [15], hDLG [16], IRF-3 [17], Bak [18], and hTERT [19]. There is also a switch from Mdm2 to HPV E6 mediated degradation of p53 in cervical cancer cells [20]. HPV16 E6 regulates cell differentiation, adhesion, polarity, proliferation, apoptosis, gene transcription, and chromosomal stability through these interactions. The interactions are not only important for the cell carcinogenesis but also for the viral survival in the host.

ING4 is one member of the inhibitor of growth (ING) family of type II tumor suppressors [21]. ING1 is the first member in this family, which plays an essential role in senescence and apoptosis [22], [23]. ING4 is located on chromosome 12p13 and encodes a 249-amino acid protein containing a highly conserved C-terminal plant homeodomain finger motif (PHD) and 2 nuclear localization signals. The PHD is also found in proteins that are associated with chromatin remodeling activities [24]. ING4 interacts with the p65 subunit of NF-kB and inhibits the transactivation of NF-kB target genes [25]. ING4 induces apoptosis through a p53 dependent pathway. The mechanism behind this manner involves increasing p53 acetylation, inhibiting Mdm2-mediated degradation of p53 and enhancing the expression of p53 responsive genes both at transcriptional and post-translational level [22], [23]. ING4 can also regulate other transcription factors, such as hypoxia-inducible factor (HIF) [26]. Although it has been demonstrated that the dysfunction of ING family proteins in many human cancers [27], [28], the deregulation of ING4 in HPV mediated cervical carcinoma is still elusive to us. Here we report that HPV16 E6 contributes to cell survival by attenuating the function of ING4 on stabilizing p53 independent of E6AP.

## Methods

### Plasmids, Antibodies, and Cell Lines

The Flag-E6 expression vector was generated by PCR cloning of the HPV16 PCDNA3-E6 cDNAs, followed by HindIII and XbaI double digestion and insertion into the HindIII and XbaI site of the pA3F vector (Sigma, St Louis, MO). Flag-E6 L50G mutant which has been reported not to bind E6AP was generated by site-directed mutagenesis (QuikChange; Stratagene) [29]. pCDNA-ING4 was used as a template to make GST tagged ING4 full-length construct and different truncates by cloning PCR-amplified fragment into modified pGEX-2T vector at EcoRI and NotI restriction sites. E6AP siRNA and control were purchased from Dharmacon RNA Technologies. Proteasome inhibitor MG132 and histone deacetylase inhibitor trichostatin A were purchased from Calbiochem (San Diego, CA).

Rabbit polyclonal antibody reactive to ING4 epitope (residues 41–80), mouse monoclonal antibody reactive to HPV16 E6 (C1P5) and goat anti-E6AP monoclonal antibody were purchased from Santa Cruz Biotechnology, Inc. (Santa Cruz, CA). Mouse monoclonal antibody reactive to flag-epitope (M2) was purchased from Sigma-Aldrich Corp. (St. Louis, MO). Mouse monoclonal antibody against Myc epitope (9E10) was purchased from Abcam (Cambridge, MA). Rabbit polyclonal antiacetylated p53 antibody at Lys 382 was purchased from Cell Signaling (Danvers, MA).

SiHa, CaSki, C33A, HEK 293T, U2OS, Saos-2 (p53^−/−^ ) and MEF (p53^−/−^Mdm2^−/−^) (ATCC, Manassas, VA, USA) cells were grown in Dulbecco’s modified Eagle’s medium (DMEM; purchased from Hyclone Logan, UT) supplemented with 10% fetal bovine serum, 50 U/ml penicillin, 50 µg/ml streptomycin, and 2 mM L-glutamine.

### Transfection, Immunoprecipitation and Western Blotting

The cells were transfected by electroporation with a Bio-Rad Gene Pulser II electroporator. Transfected cells were harvested, washed with ice-cold PBS, and lysed in 0.5 ml ice-cold radioimmunoprecipitation buffer, supplemented with protease inhibitors. Cell debris was removed by centrifugation, lysates were then precleared by end-over-end rotation with normal mouse serum and 30 µl of a 1∶1 mixture of protein A-protein G-conjugated Sepharose beads (1 h, 4°C). Approximately 5% of the lysate was saved for input control. The protein of interest was captured by rotating the remaining lysate with 1 µg of appropriate antibody overnight at 4°C. Immune complexes were captured with 30 µl of a 1∶1 mixture of protein A and protein G Sepharose beads. For sequential immunoprecipitation assay, cell lysates were immunoprecipitated with Ezview™ Red anti-Flag M2 Affinity Gel. Flag-HPV16 E6 and the associated proteins were eluted with 3XFlag peptide. Twenty percent of the eluent was subject to Western analysis using the indicated antibodies. The remaining eluent was used for secondary immunoprecipitation with anti-Myc antibody. For Western blot assays, input lysates and immunoprecipitated (IP) complexes were boiled in Laemmli buffer, fractionated by SDS-PAGE, and transferred to a 0.45 µm nitrocellulose membrane. The membranes were then probed with appropriate antibodies followed by incubation with appropriate infrared-tagged secondary antibodies and viewed on an Odyssey imager (LiCor Inc., Lincoln, NE).

### GST Fusion Protein Purification and GST Pull-down Assay

Escherichia coli BL21 (DE3) cells were transformed with the plasmid constructs for each GST fusion protein. Single colonies were picked and grown overnight in 3 ml of Luria broth supplemented with 100 µg/ml ampicillin. One milliliter of the overnight culture was used to inoculate a 500 ml culture. The larger culture was incubated until the optical density at 600 nm was approximately 0.6, at which point it was induced with 1 mM isopropyl-β-D-thiogalactopyranoside (IPTG) for 12 h at 30°C. The bacteria were pelleted, washed once with STE buffer (100 mM NaCl, 10 mM Tris, and 1 mM EDTA, pH 7.5), resuspended in 3 ml NETN buffer (0.5% NP-40, 100 mM NaCl, 20 mM Tris, 1 mM EDTA, pH 8.0), supplemented with protease inhibitors, and incubated on ice for 15 min. A volume of 150 µl of 1 M dithiothreitol (DTT) and 1.8 ml of a 10% solution of Sarkosyl in STE buffer was added, and the suspension was sonicated (for 3 min on ice) to solubilize the proteins. The lysates were centrifuged (12,000×g, 10 min, 4°C) to separate the unsolubilized fraction. The clear supernatant was transferred to a fresh tube, to which 3 ml of 10% Triton X-100 in STE buffer and 200 µl of Glutathione-Sepharose beads were added. The tube was rotated overnight at 4°C, after which the purified protein bound to Glutathione was collected by centrifugation (2 min, 600×g, 4°C) and washed five times with NETN buffer supplemented with protease inhibitors. The level of purification was determined by SDS-PAGE, and purified proteins were stored at 4°C. For pull-down assays from cell lysates, lysates were prepared in RIPA buffer (0.5% NP-40, 10 mM Tris [pH 7.5], 2 mM EDTA, 150 mM NaCl, supplemented with protease inhibitors). Lysates were precleared and then rotated with either GST control or the appropriate GST fusion protein bound to Glutathione-Sepharose beads. For in vitro binding experiments, GST fusion proteins were incubated with ^35^S-labeled in vitro-translated protein in binding buffer (1x PBS, 0.1% NP-40, 0.5 mM DTT, 10% glycerol, supplemented with protease inhibitors). In vitro translation was performed with the T7-TNT Quick Coupled transcription-translation system (Promega Inc.,Madison, WI) according to the manufacturer’s instructions.

### Immunofluorescence

To check the co-localization ectopically expressed Flag-E6 and PCDNA-ING4 in the cells, we used Lipofectamine 2000 (Invitrogen, Carlsbad, CA) to transfect Saos2 cells with the plasmids then cultured on coverslips. At 36 h posttransfection, cells were fixed using 3% paraformaldelhyde with 0.1% Triton X-100 for 20 min at room temperature. We used CaSki cells to examine the co-localization of endogenous E6 with ING4, transferred appropriate CaSki cells onto slides and fixed them using the same method as above after culture for 5 hours. Fixed cells were washed with PBS and subsequently blocked in 1% BSA for 10 min. ING4 was detected using rabbit polyclonal antibody reactive to ING4. Endogenous E6 was detected using E6-reactive mouse monoclonal antibody (1∶150 dilution); Flag-tagged E6 was detected using M2 antibody (1∶1,000 dilution; Santa Cruz Biotechnology, Inc., Santa Cruz, CA). Primary antibodies were incubated with the cells for 30 min at RT. Cells were washed three times with PBS and exposed to secondary antibodies. Goat anti-mouse antibody conjugated to Alexa Fluor 594 detecting E6 and goat anti-rabbit antibody conjugated to Alexa Fluor 488 detecting ING4 were used as secondary antibodies respectively. Secondary antibodies were diluted in blocking buffer at 1∶1,000 and incubated for 1 h at RT, followed by three washes with blocking buffer. The last wash contained 4′, 6′-diamidino-2-phenylindole (DAPI; Promega, Madison, WI) to counterstain the nuclei. The slides were examined using Olympus confocal microscopy and the images were analyzed with a Fluoview FV300 (Olympus, Melville, NY) software.

### Luciferase Reporter Assay

Twelve million cells were co-transfected by using a Bio-Rad electroporater (Bio-Rad Laboratories, Inc., Hercules, CA) with 2 µg p21^WAF1/CIP1^ reporter construct with combinations of different plasmids. At 24 hours post-transfection, cells were harvested, washed in PBS, and lysed in cell lysis buffer (BioVision, Inc., Mountain View, CA). Fifty microliter of cell lysate was used for the reporter assay, using an LMaxII384 luminometer (Molecular Devices, Inc., Sunnyvale, CA). A portion of the cell lysate was used for Western blotting. Transferred proteins were detected with Odyssey infrared scanning technology (LI-COR, Inc., Lincoln, NE), using Alexa Fluor 680 and Alexa Fluor 800 (Molecular Probes, Carlsbad, CA, and Rockland, Gilbertsville, PA, respectively). The results are shown as the means of the data from three independent experiments.

### E6AP siRNA and Lentiviral-mediated HPV16 E6 Gene Silencing

The human E6AP small interfering RNA oligo was purchased from Dharmacon (Chicago,IL). The sequence for its sense oligo is 5′-CUUUCUCAAUGCACUUG UAUU-3′. Transfection of E6AP small interfering RNA into U2OS cells was done using a Lipofectamine 2000 kit (Invitrogen) according to the manufacturer’s instructions.

For the lentivirus-mediated stable knock down of HPV16 E6, the E6 shRNA sequence (5′-GGACAGAGCCCATTACAATAT-3′) was inserted into pGIPZ vector according to the manufacture’s instructions (Open Biosystem, Inc, Huntsville, AL), the vector expressing HPV16 E6 small hairpin RNA was abbreviated as sh-E6. In addition, a 21-mer oligonucleotide (TCTCGCTTGGGCGAGAGTAAG) that had no significant homology to any known human mRNA in the databases was cloned in the same vector and used as control. Control shRNA is hereinafter abbreviated as sh-C.

Lentiviruses were produced by transient transfection into HEK 293T cells, a total of 2×10^6^ HEK 293T cells were seeded in 10-cm-diameter dishes in DMEM (HyClone, Logan, UT) supplemented with 10% FBS and 1% antibiotic-antimycotic and cultured in a 5% CO_2_ incubator for 24 h prior to transfection. A total of 20 µg of plasmid DNA was used for the transfection of each dish, including 1.5 µg of envelope plasmid pCMV-VSV-G (catalog no.8454;Addgene, Inc., Cambridge, MA), 3 µg of packaging plasmid pRSV-REV (catalog no. 12251 Addgene, Inc., Cambridge, MA), 5 µg of packaging plasmid pMDLg/Prre (catalog no. 12251 Addgene, Inc., Cambridge, MA), and 10.5 µg of lentiviral vector plasmid. The precipitation was formed by adding the plasmids to a final volume of 438 µl of H_2_0 and 62 µl of 2 M Cacl_2_, mixing well, adding 500 µl of 2×HEPES-buffered saline, and then incubating at room temperature for 30 min. Chloroquine was added to the 10 ml of plated media with a final concentration of 25 µM at 5 minutes prior to transfection. The medium was replaced after 12 h with DMEM supplemented with 10% FBS and 10 mM HEPES, and 10 mM sodium butyrate. The medium was replaced again 10 hours later using DMEM supplemented with 10% FBS and 10 mM HEPES. The conditioned medium was collected four times at 12 h interval, filtered through 0.45 µm pore-size cellulose acetate filters, and stored on ice. The virus was concentrated by spinning at 70,000×g for 2.5 h. The concentrated virus was resuspended in RPMI then used to infect 10^6^ cells in the presence of 20 µM/ml Polybrene. After 72 h, puromycin was added to final concentration of 2 µg/ml for selection. GFP immunofluorescence was assessed by using an Olympus IX71 microscope filtered with 560-nm excitation and 645-nm emission filters. The cells were grown to 80% confluence in the presence of 2 µg/ml puromycin prior to Western blot.

### Colony Formation Assay

Ten million of Saos-2 cells were typically transfected using electroporation with different combinations of expression plasmids as shown in the text. Transfected cells were cultured in the selection medium (Dulbecco’s modified Eagle’s medium [DMEM] supplemented with 5 mg/ml G418). After a 2-week selection, cells were fixed on the plates with 4% formaldehyde and stained with 0.1% crystal violet. The amount of the colonies in each dish was scanned by Li-Cor Odyssey and counted. The data are presented as the average from two independent experiments.

### Apoptosis Assay

The transfected cells were analyzed by propidium iodide (PI) flow cytometric assay, which is based on the principle that apoptotic cells are characterized by DNA fragmentation and the consequent loss of nuclear DNA content at the late phase of apoptosis. Briefly, 10^6^ cells were washed with PBS and fixed with 100% ethanol 30 min at 4°C. The fixed cells were then stained with 50 µg/ml of PI (Sigma, St. Louis, MO) with 1 µg/ml RNase at 4°C for 1 hour. PI binds to DNA by intercalating between the bases without sequence preference. Different cell cycle phases were characterized by their different DNA contents by using a FACSCalibur cytometer (Becton Dickinson, San Jose, CA), and the results were analyzed by FlowJo Software (Tree Star, Ashland, OR).

## Results

### HPV16 E6 Forms Complex with ING4 Independent of p53

It has been showed that HPV16 E6 forms complex with tumor-suppressor protein p53 by recruiting the cellular ubiquitin–protein ligase E6-AP for ubiquitin–proteasome-mediated degradation [5], [6]. Other pathways and mechanisms by which HPV16 E6 may regulate p53 function still need to be elucidated. ING4 has been proved to interact with p53 and enhance its activity [21]. Now we want to see whether HPV16 E6 contributes to cell survival by inhibiting ING4 function on p53. First we investigated whether HPV16 E6 forms a complex with ING4 in cervical carcinoma cells. Endogenously expressed HPV16 E6 was immunoprecipitated from HPV16 positive cervical carcinoma cells (CaSki and Siha), the co-immunoprecipitation (IP) of ING4 was monitored by the polyclonal antibody reactive to ING4, HPV negative cervical carcinoma cell line C33A was used as a negative control. The result showed that HPV16 E6 formed stable complex with ING4 (Fig. 1A). In order to confirm the possibility that HPV16 E6 combines with ING4 without p53 introduction, p53 null cell line Saos2 was contransfected with constructs expressing Flag tagged HPV16 E6 and pCDNA-ING4, empty vector was used as a control. Whole-cell extracts of the transfected Saos2 cells were precipitated with anti-ING4 antibody, and the precipitates were analyzed by Western blotted with anti-Flag antibody. Transfected HPV16 E6 and pCDNA-ING4 also formed complex independent of p53 (Fig. 1B). We also performed in vitro binding assay to determine whether HPV16 E6 directly interacts with ING4. The GST-ING4 and GST expression constructs were bacterially expressed and incubated with in vitro translated ^35^S-labeled HPV16 E6, and the pull-down result showed that GST-ING4 beads but not GST alone precipitated a significant amount of HPV16 E6 protein with radioactivity. Former studies showed that the NLS domain of ING4 is responsible for combining with p53, in order to map the combining domain of ING4 with HPV16 E6, a series of GST-tagged ING4 truncates were generated to pull-down ^35^S-radiolabeled in vitro translated HPV16 E6 protein. The result indicated that full-length ING4 and NLS domain containing region 120–184 combined with HPV16 E6. The amount of GST and GST-ING4 proteins used in the binding assay was showed by Coomassie blue stained gels (Fig. 1C and D). So ING4 may have a common binding region for both p53 and HPV16 E6. Then we have reason to imagine that there is a competition relationship between p53 and HPV16 E6 for binding with ING4. We conclude that HPV16 E6 and ING4 form complex both in vivo and in vitro. The interaction of HPV16 E6 and ING4 was further examined by immunostaining assays. Ectopically expressed PCDNA-ING4 and Flag-E6 co-localized to the nucleus of SaoS2 cells (Fig. 1E). Similarly, endogenous E6 accumulated in the nucleus of CaSki cells co-localized with endogenous ING4 (Fig. 1F).

**Figure 1:** HPV16 E6 forms complex with ING4 independent of p53. (A) Lysates from HPV negative cervical carcinoma cell line C33A and two HPV16 positive cell lines CaSki and SiHa were subjected to IP with HPV16 E6 specific antibody C1P5 and detected by Western blotting (WB) for the indicated proteins. (B) Saos2 cells were co-transfected with Flag-tagged E6 and PCDNA-ING4, balanced with empty vector. The cell lydates were subjected to IP with ING4 specific antibody and detected by WB. (C) and (D) Either GST control, GST-ING4 full length or truncates beads were incubated with HPV16 E6 in vitro translated protein with ^35^S-radiolabeled. 5% of in vitro translated protein input was used as a comparison. Precipitated proteins were resolved by SDS-PAGE, exposed to phosphorimager screen and scanned by Typhoon 9410 imaging system. Coomassie blue staining of SDS-PAGE-resolved purified GST and GST-ING4 proteins was shown under the panel. (E) Colocalization of ectopically expressed ING4 and HPV16 E6. Saos2 cells plated on coverslips were transfected with Flag-E6 and PCDNA-ING4 using Lipofectamine 2000. (F) Colocalization of endogenous HPV16 E6 and ING4 in CaSki cells. All panels are representative pictures from approximately 50 cells of five different fields of three independent experiments.

### p53 Binding to ING4 and Acetylation was Attenuated by HPV16 E6

Despite HPV16 E6 interacted with ING4, we did not find HPV16 E6 inhibited ING4 stability (Fig. 2A ). Then we looked into the possibility that HPV16 E6 might attenuate p53 function through hindering the association of ING4 and p53 besides p53 degradation. We first examined possibility that there was a cross connection among HPV16 E6, p53 and ING4 by a sequential immunoprecipitation assay. These three proteins were co-expressed in p53^−/−^Mdm^−/−^ MEF cells. An initial immunoprecipitation assay using an anti-Flag antibody against Flag-E6 pulled down both ING4 and Myc-53 (Fig. 2B, lane 4). The immunocomplexes were eluted and Myc-p53 was subsequently precipitated by an anti-Myc. Flag-E6 and ING4 were present in the anti-Myc-p53 precipitates (Fig. 2B, lane 6), indicating that these three proteins combine each other. Then we tested whether HPV16 E6 affected ING4 and p53 interaction. ING4 and p53 both were expressed in p53^−/−^Mdm^−/−^ MEF cells with or without HPV16 E6. To rule out the possibility that the diminished p53-ING4 association is caused by p53 protein degradation, we treated transfected cells with the proteasome inhibitor MG132 to block protein degradation, thus equalizing the ING4 and p53 protein levels among cell groups, the ING4-p53 interaction was significantly weakened in a dose-dependent manner when HPV16 E6 increased (Fig. 2C). To further confirm that less ING4 combined with p53 when HPV16 E6 exits, we reciprocally knockdown HPV16 E6 level in CaSki and SiHa cells by transduction with shRNA-containing lentivirus and made stable cell lines carrying the sh-E6 vector and the sh-control vector by selection. The whole cell lysates of the above cells were immunoprecipitated with anti-p53 antibody and analyzed the combined ING4 by Western blot. The result showed that the amount of precipitated ING4 was much more elevated comparing with the increasing amount of p53 in HPV16 E6 knock-down cells. This phenomenon further proved that there was more ING4 protein combined with p53 when HPV16 E6 was down-regulated (Fig. 2D). Since the stoichiometry of in vivo p53-ING4 complexes is not known, and both p53 and ING4 likely form many other complexes with other proteins. To prove HPV16 E6 attenuates ING4 and p53 association independent of p53 degradation, we co-transfected pCDNA-ING4, Myc-p53 and flag-tagged HPV16 E6 or it’s mutant L50G which has been showed defective in binding with E6AP and p53 degradation into Saos2 cell [29]. Immunoprecipitation with Flag antibody M2 showed that E6AP binding defective HPV16 E6 L50G combined with ING4. The amount of ING4 binding with p53 was diminished both with wild type HPV16 E6 and mutant HPV16 E6 L50G (Fig. 2E). So the recruitment of E6AP for p53 degradation is not necessary for disturbing the binding of ING4 and p53 by HPV16 E6. ING4 is believed to be involved in regulating p53 function by acetylation on Lys-382. To determine whether ING4 mediated p53 acetylation is attenuated by HPV16 E6, we co-transfected PCDNA-ING4 and Myc-p53 into SaoS2 cell in the presence of Flag tagged HPV16 E6 or its mutant L50G. At 24 hours post-transfection, histone deacetylase inhibitor trichostatin A were added for additional 6 hours before harvest to stabilize acetylated p53. HPV16 E6L50G did not bind with E6AP and had little role on p53 degradation, ING4 binding with p53 was attenuated and its induced p53 acetylation was nearly nullified when HPV16 E6 or its mutant L50G exited (Fig. 2E). An in vitro GST assay using recombinant purified protein also indicated that HPV16 E6 attenuated the interaction between ING4 and p53 (Fig. 2F).

**Figure 2:** HPV16 E6 binds to ING4 and hinders its association with p53. (A) HPV16 E6 does not affect ING4 stability. p53^−/−^Mdm2^−/−^MEF cells were transfected with ING4 and an increasing amount of either Flag-HPV16 E6 or control vector. The levels of ING4, HPV16 E6 and GAPDH were examined by Western blot. (B) HPV16 E6, ING4 and p53 bind each other. Flag-E6, PCDNA-ING4, and Myc-p53 were transfected into p53^−/−^Mdm2^−/−^MEF cells. Cell lysates were immunoprecipitated with EzviewTM Red anti-Flag M2 Affinity Gel (lanes 3 and 4), Flag-E6 and the associated proteins were eluted with 3XFlag peptide. Twenty percent of the eluent was subject to Western analysis using indicated antibodies. The remaining eluent was used for secondary immunoprecipitation with anti-myc antibody (lanes 5and 6). (C) Saos2 cells were transfected with PCDNA-ING4, Myc-p53, and either increasing amounts of HPV16 E6 or the vector control. Transfected cells were treated with MG132 for 6 h. The association of PCDNA-ING4 and Myc-p53 was analyzed by immunoprecipitation assay with anti-p53 antibody. (D) Knockdown of HPV16 E6 increases the ING4-p53 interaction. CaSki and SiHa cells with lentivirus-delivered GFP labeled shRNA against HPV16 E6 (shE6) or scramble control (shC) were shown on the left panel. On the other side, the top panel showed the whole cell lysates were immunoprecipitated with anti-p53 antibody and checked ING4 expression by Western blot. Input equivalent to 10% of the whole cell lysates used for immunoprecipitation was subjected to Western blot using the indicated antibody. (E) ING4 mediated p53 acetylation was attenuated by HPV16 E6. Saos2 cells were transfected with PCDNA-ING4, Myc-p53, in the present of either HPV16 E6 or its mutant L50G. At 24 hr post transfection, trichostatin A were added for additional 6 hours, immunoprecipitation and western blot showed that HPV16 E6L50G attenuated binding and acetylation induced by ING4 on p53 without p53 degradation mediated by E6AP. (F) HPV16 E6 attenuates the binding affinity between ING4 and p53 in vitro. Myc-tagged p53 was incubated with bacterially-expressed GST or GST-ING4 in the presence of Flag-tagged HPV16 E6 or control vector for GST-pull down assay. Concentration of each fusion protein used in GST-pull down assays was kept the same. The level of myc-p53 pulled down by GST-ING4 was less in the presence of HPV16 E6.

### ING4 Function on p53 was Diminished when HPV16 E6 Existed

ING4 enhances p53 acetylation and activates p53 mediated p21 promoter [21]. HPV16 E6 switches p53 degradation from Mdm2 pathway to E6 mediated pathway [20]. Therefore, in order to further determine whether HPV16 E6 attenuates ING4 enhancing role on p53 transcriptional activity, we performed reporter assay by co-transfected p21^WAF1/CIP1^ reporter construct with combinations of different plasmids into Saos-2 cells. The result showed that both HPV16 E6 and its mutant L50G diminished the transcriptional activity of p53 in the present of ING4, the expression levels of p53, ING4, E6 and GAPDH as a loading control, were also analyzed by western blot. (Fig. 3A). While it has been showed that HPV16 E6 L50G did not bind to E6AP nor cause p53 degradation, we can conclude that HPV16 E6 may attenuate ING4 enhancing role on p53 independent of its degradation. Previous studies have showed that ING4 inhibits cell growth and leads to apoptosis in a p53-dependent manner [21]. We used colony formation assay to check the effect of HPV16 E6 and its mutant L50G on p53 as well as ING4 mediated cell apoptosis. The results showed that co-expression of ING4 with p53 markedly decreased the colony formation of Saos-2 cell compared to that produced by p53 alone. So ING4 significantly enhanced the blocking ability of p53 on colony formation; Wild-type HPV16 E6 reverse this kind of blocking role of p53 and ING4, while HPV16 E6L50G nullified the p53 role mainly when ING4 existed. (Fig. 3B). HPV16 E6 blocks apoptosis by recruiting the cellular ubiquitin-protein ligase E6AP to target p53 for degradation [5]. To further determine whether HPV16 E6 can diminish ING4 triggering apoptosis besides direct p53 degradation, U2OS cells were transfected with siRNA Luciferase or siRNA E6AP combined with ING4 or ING4 plus HPV16 E6. The E6AP expression was significantly knocked down in cells transfected with siRNA E6AP compared to siRNA Luciferase control. The levels of cells undergoing apoptosis (sub-G_1_ phase) were examined. The apoptosis rate in ING4 transfected cells is approximately 6 times higher than transfected with only control vectors in the Lucifersase knock-down cells; ING induced apoptosis increased nearly 5 times in the E6AP knock-down cells. However, the ING4 induced p53-mediated apoptosis was obviously decreased when co-transfected with HPV16 E6 even in the E6AP knock-down cells (Fig. 4C). These results consistently confirmed that ING4 mediated p53-dependent apoptosis could be blocked by HPV16 E6 independently of p53 degradation.

**Figure 3:** HPV16 E6 suppresses the ING4 mediated p53 transcriptional activity and apoptosis. (A ) Saos-2 (p53^−/−^) cells were cotransfected with a wild-type p21WAF1/CIP1 promoter construct, different combinations of plasmids expressing Myc-p53, PCDNA-ING4, flag-tagged HPV16 E6 or its mutant L50G. At 36 h posttransfection, cells were harvested and lysed in reporter lysis buffer. The bars plot the means of the results of two independent experiments. Error bars represent standard deviations (SD). The results showed that HPV16 E6 attenuates ING4-triggered p53 transcriptional activity. The expression levels of each target proteins were detected by western blotting and shown at the bottom panels. (B) Saos2 cells were transfected with expression plasmids for myc-p53, PCDNA-ING4, in combinations with flag-E6 or its mutant L50G. After a 2-week selection, cells were fixed on the plates with 4% formaldehyde and stained with 0.1% crystal violet. A representative of colony formation was shown. The area of colonies (pixels) in each dish was calculated by Li-Cor Odyssey. The number represents the averages of data from two independent experiments.

**Figure 4:** HPV16 E6 suppresses the ING4 mediated p53 transcriptional activity and apoptosis. (C) U2OS cells were respectively transfected with siRNA Luciferase or siRNA E6AP, with ING4 or ING4+E6 using the Lipofectamin 2000. Cells were collected at 36 h posttransfection after a 12-h serum starvation and fixed. Levels of cells undergoing apoptosis (sub-G1 phase) in individual PI-stained samples were analyzed by flow cytometry, and the data were analyzed by FlowJo software. The bar diagram represents the mean of three independent experiments. Western blot showing the protein level of E6AP in the lentivirus-mediated E6AP of control knockdown cell lines. GAPDH was used as the loading control.

## Discussion

The inhibitor of growth (ING) family is reported to be involved in apoptosis, cell cycle and DNA repair. Their expression is down-regulated in several cancer types, but they are rarely mutated in human cancer [22, 23, 27, and 30]. ING4, as a member of ING family, binds to p53 and modulates its transcriptional activity [21]. One important genetic alteration in a variety of human cancer is the inactivation of the tumor suppressor function in p53. HPV oncogenic protein E6 is an important carcinogenic agent in cervical cancer [4]. HPV E6 promotes cell proliferation through intervening in functions of several cellular agents by protein-protein interactions. One fundamental mechanism for HPV E6 contributes to cell proliferation is that HPV E6 recruits E6-AP in stimulating the degradation of p53 via ubiquitin-dependent proteolytic system [5], [6]. However HPV E6 can also contribute cell transformation without p53 degradation [31]. Because both ING4 and HPV16 E6 are known to regulate p53 function, we have reason to characterize in more detail the putative physical and functional interaction between ING4 and HPV16 E6.

First we confirmed that ING4 and HPV16 E6 bind each other in vivo and in vitro independently of p53 introduction. Like other members in the ING family, ING4 contains several highly conserved domains, including a leucine zipper-like motif, two nuclear localization signal domains (NLS1 and NLS2), and a C-terminal plant homeodomain (PHD). Our results showed that ING4 combines with HPV16 E6 through its NLS domain which sharing a common region binding with p53. The NLS region is essential for the subnuclear localization of ING4 and its relationships with p53 [32], [33]. Through this binding ING4 functionally enhanced acetylaiton of p53 on Lys-382 and up-regulated its transcriptional activity. It is has been reported that the acetylation of p53 lys-382 is an important regulation event in cell apoptotic pathway [34]. Next we investigated whether ING4 association with p53 and its function in stabilizing p53 was attenuated when HPV16 E6 existed. We determined that ING4, HPV16 E6 and p53 form a ternary complex through a sequential immunoprecipitation. To test the effect of HPV16 E6 on the relationship of ING4 and p53, at the same time excluding direct p53 degradation impact, we immunoprecipitated ING4 and checked p53 protein level with increasing HPV16 E6 amount in the presence of proteasome inhibitor MG132. Competitive binding and in vitro binding assays showed that the amount of p53 combined with ING4 became less when HPV16 E6 protein expressed. HPV16 E6 mutant L50G defective in binding with E6AP nor causing p53 degradation also has the ability inhibiting the interaction of ING4 and p53 as well as p53 acetylation. ING4 has been reported to up-regulate p53 activity by enhancing p53 acetylation via recruiting p300 [21]. The interaction with p300 is also necessary for E6 to inhibit p53 dependent chromatin transcription and p300 mediated p53 acetylation. E6 mutant defective in inducing p53 degradation remains this ability and E6AP is not required for E6-p53-p300 complex formation [29], [35], [36]. At last, functional analysis revealed that HPV16 E6 attenuated ING4 triggered p53 mediated apoptosis besides directly causing p53 degradation. In spite of that inducing p53 degradation is an important function of the E6 protein, the analysis of E6 mutants and E6AP null cell demonstrates that other activities are required for its oncogenical transformation [37]. Our results indicate HPV16 E6 attenuates ING4 role on p53 stabilizing independently of p53 degradation. One mechanism behind these phenomena is that the binding activity among these three proteins has a competitive relationship for they share a common combining domain. ING4 enhances acetylation of p53 on Lys382 and upregulates p53 transcriptional activity [21]. Acetylation of p53 at several C-terminal lysine residues may attribute its function by increasing p53’s DNA binding capacity, target gene selectivity and transcription-activating properties [38]. Blocking ING4 mediated p53 acetylation by HPV16 E6 may provide a new mechanism for HPV as far as other tumor virus induced cell carcinogenesis [28]. High risk HPVs play a pivotal role in the development of cervical carcinoma.

### Conclusions

ING4 binding with p53 and induced p53 acetylation as well as its triggered p53 mediated apoptosis were attenuated by HPV16 E6 independent of p53 degradation.
